The article "Function and regulation of transforming growth factor β1 signalling in antler chondrocyte proliferation and differentiation" was published in 2019. Journal: Cell Prolif.

# Function and regulation of transforming growth factor β1 signalling in antler chondrocyte proliferation and differentiation

**DOI:** 10.1111/cpr.12637

**Published:** 2019-06-06

**Authors:** Li Ma, Zhan‐Qing Yang, Jun‐Li Ding, Shu Liu, Bin Guo, Zhan‐Peng Yue

**Affiliations:** ^1^ College of Veterinary Medicine Jilin University Changchun China

**Keywords:** antler chondrocyte, Foxa, Notch and Shh signalling, proliferation and differentiation, TGFβ1 signalling

## Abstract

**Objectives:**

Chondrocyte proliferation and differentiation are crucial for endochondral ossification, but their regulatory mechanism remains unclear. The present study aimed to determine the physiological function of TGFβ1 signalling in the proliferation and differentiation of antler chondrocytes and explore its relationship with Notch, Shh signalling and Foxa.

**Materials and methods:**

Immunofluorescence, Western blot, MTS assay, flow cytometry, RNA interference and real‐time PCR were used to analyse the function and regulatory mechanisms of TGFβ1 signalling in antler chondrocyte proliferation and differentiation.

**Results:**

TGFβ1, TGFBR1 and TGFBR2 were highly expressed in antler cartilage. TGFβ1 promoted chondrocyte proliferation, increased the proportion of S‐phase cells and induced the expression of hypertrophic chondrocyte markers Col X, Runx2 and Alpl. However, this induction was weakened by TGFβ receptor inhibitor SB431542 and Smad3 inhibitor SIS3. Simultaneously, TGFβ1 activated Notch and Shh signalling whose blockage attenuated the above effects of rTGFβ1, whereas addition of rShh rescued the defects in chondrocyte proliferation and differentiation elicited by SB431542 and SIS3. Further analysis revealed that inhibition of Notch signalling impeded TGFβ1 activation of the Shh pathway. Knockdown of Foxa1, Foxa2 and Foxa3 abrogated the effects of TGFβ1 on chondrocyte differentiation. Notch and Shh signalling mediated the regulation of Foxa transcription factors by TGFβ1.

**Conclusions:**

TGFβ1 signalling could induce the proliferation and differentiation of antler chondrocytes through Notch‐Shh‐Foxa pathway.

## 1 INTRODUCTION

Chondrocyte proliferation and differentiation are two key processes in cartilage ossification.^1^ As a bone organ, antler growth involves the rapid proliferation of chondrocytes, without becoming cancerous, and then differentiation into hypertrophic chondrocytes. Thus, this is a good model for exploring the mechanisms of cartilage and bone development.^2^

Transforming growth factor beta (TGFβ) superfamily member TGFβ1, a regulator of cell proliferation and differentiation in many biological processes, is expressed abundantly in bone and plays an important role in bone physiology and homeostasis.^3^, ^4^ Ablation of TGFβ1 led to visibly decreased longitudinal long bone growth along with reduced hypertrophic chondrocyte numbers.^5^ Further analysis shows that TGFβ1 may bind to the TGFβ1 type II receptor (TGFΒR2) and activates the type I transmembrane serine/threonine kinase receptor (TGFΒR1), leading to the phosphorylation of Smad transcription factors, which serve as the principal facilitators of TGFβ signalling.^6^, ^7^ Conditional knockout of TGFΒR2 or mutant of Smad3 exon 8 resulted in the degenerative joint disease and progressive osteoarthritis‐like phenotype accompanied by the aberrant chondrocyte proliferation and differentiation.^8^, ^9^, ^10^, ^11^ Silencing of Smad3 impeded the TGFβ‐induced chondrogenic differentiation.^12^ However, few studies have reported the physiological function of TGFβ1 signalling in antler chondrocyte proliferation and differentiation.

The article "Function and regulation of transforming growth factor β1 signalling in antler chondrocyte proliferation and differentiation" was published in 2019. Journal: Cell Prolif.

Notch signalling is critical for cartilage development and endochondral ossification.^13^, ^14^, ^15^, ^16^ Blockage of Notch signalling delayed chondrocyte maturation and suppressed chondrocyte proliferation, whereas activation of Notch signalling promoted chondrocyte hypertrophy.^14^, ^15^, ^16^ Further studies demonstrated that Sonic hedgehog (Shh) signalling acted downstream of Notch pathway to mediate the proliferation and differentiation of antler chondrocytes.^17^ In rat mesenchymal stem cells (MSCs), TGFβ1 could affect the expression of Shh and Gli1,^18^ but the relationship among TGFβ1, Notch and Shh signalling in chondrocyte proliferation and differentiation remains unknown. It has been previously reported that Foxa transcription factors are key regulators of chondrocyte differentiation. Chondrocyte‐specific knockout of Foxa2 and Foxa3 led to post‐natal dwarfism with profound defects in chondrocyte hypertrophy and mineralization in the sternebrae.^19^ However, little is known whether Foxa may mediate the effects of TGFβ1 signalling on chondrocyte proliferation and differentiation.

In this study, we investigated the function of TGFβ1 signalling in the proliferation and differentiation of antler chondrocytes and explored its relationship with Notch, Shh signalling and Foxa. The results evidenced that TGFβ1 signalling might induce the proliferation and differentiation of antler chondrocytes through activating Notch‐Shh‐Foxa pathway.

## 2 MATERIALS AND METHODS

### 2.1 Tissue collection

Antler tissues were collected from 3‐year‐old healthy sika deer as previously described.^20^ The distal 5 cm of growing tip was removed and sectioned sagittally along the longitudinal axis. A part of the tip was then cut into 4‐6 mm pieces, flash frozen in liquid nitrogen and stored at −80°C for immunofluorescence, and the remaining tip was used for isolation of antler chondrocytes.

The article "Function and regulation of transforming growth factor β1 signalling in antler chondrocyte proliferation and differentiation" was published in 2019. Journal: Cell Prolif.

### 2.2 Antler chondrocyte treatment

Antler chondrocytes were isolated by enzymatic digestion as previously described^20^ and cultured with DMEM‐high glucose (Hyclone) supplemented with 10% foetal bovine serum (Life Technologies). These cultured chondrocytes were treated with recombinant human/mouse/rat TGFβ1 protein (rTGFβ1, 100 ng/mL; R&D Systems) in the absence or presence of TGFβ receptor inhibitor SB431542 (10 µmol/L, MCE), Smad3 inhibitor SIS3 (10 µmol/L; Selleck), Notch signalling inhibitor DAPT (25 µmol/L; Sigma), Smo antagonist cyclopamine (10 µmol/L; Tocris Bioscience) and Gli1 antagonist GANT58 (10 µmol/L; Tocris Bioscience), respectively. Additionally, chondrocytes were incubated with SB431542 or SIS3 and then supplemented recombinant human Shh protein (rShh, 25 ng/mL; R&D Systems).

### 2.3 Immunofluorescence

Frozen antler cartilage sections were fixed in 4% paraformaldehyde solution for 30 minutes and then washed three times with PBS and blocked with 3% BSA for 2 hours. After incubation with primary antibody TGFβ1 (1:200; Abcam), TGFBR1 (1:500; Abcam) or TGFBR2 (1:200; Abcam) overnight at 4°C, these sections were washed and then treated with Alexa Fluor Plus 488 goat anti‐rabbit IgG secondary antibody (Invitrogen) for 1 hour. Nuclei were stained with DAPI. Fluorescent signals were examined under a fluorescence microscope.

### 2.4 Western blot

Western blot was performed according to an existing research method,^21^ and cells were lysed using protein lysate. The entire protein was then transferred onto PVDF membranes. After blocking with 5% non‐fat milk, the membranes were probed with Smad3 (1:5000; Abcam) and p‐Smad3 (1:5000; Abcam) antibodies, washed with PBS and then incubated with HRP‐linked secondary antibodies. Bands were visualized with an enhanced chemiluminescence substrate (Thermo Fischer Scientific). β‐actin was used to normalize the protein levels.

### 2.5 MTS assay

Cell proliferation was analysed using MTS assay (Promega) in accordance with the manufacturer's protocol. Briefly, antler chondrocytes were treated as described above, at which time 20 µL of MTS reagent was added to each well and incubated for 4 hours. The absorbance was measured at 490 nm using a 96‐well plate reader. Each experiment was performed in triplicate.

### 2.6 Flow cytometry

After antler chondrocytes were synchronized by serum starvation, they were treated as described above. Cells were harvested by trypsinization and centrifugation, washed with PBS and then fixed overnight at 4°C in 70% ethanol. The fixed cells were washed with PBS and stained with 0.5 mL PI/RNase staining buffer (BD Biosciences) for 15 minutes at room temperature. Then, the stained cells were analysed by flow cytometry.

The article "Function and regulation of transforming growth factor β1 signalling in antler chondrocyte proliferation and differentiation" was published in 2019. Journal: Cell Prolif.

### 2.7 RNA interference

Small interfering RNA (siRNA) for targeting Shh, Gli1, Gli2, Gli3, Foxa1, Foxa2 and Foxa3 as well as a scrambled siRNA (negative control) were designed and synthesized by GenePharma, and the corresponding sequences are listed in Table 1. Transfection for siRNA was performed according to Lipofectamine 2000 protocol (Invitrogen). After transfection with the corresponding siRNA, antler chondrocytes were collected for 24 hours in the absence or presence of rTGFβ1 and rShh, respectively.

**Table 1:** The siRNAs used in this study

Gene	Sense	Antisense
Shh	GCACCAUUCUCAUCAACCGTT	CGGUUGAUGAGAAUGGUGCTT
Gli1	GCAGCUUGUGUGUAAUUAUTT	AUAAUUACACACAAGCUGCTT
Gli2	GGCUGAGGUGGUCAUCUAUTT	AUAGAUGACCACCUCAGCCTT
Gli3	CCACUUCCAAUGAUUCUUUTT	AAAGAAUCAUUGGAAGUGGTT
Foxa1	GGUCUGGGCACCAUGAAUUTT	AAUUCCAUGGUGCCCAGACCTT
Foxa2	CCCUACGCGAACAUGAACUTT	AGUUCAUGUUCGCGUAGGGTT
Foxa3	UCCUACAUCUCGCUCAUCATT	UGAUGAGCGAGAUGUAGGATT
Negative Control	UUCUCCGAACGUGUCACGUTT	ACGUGACACGUUCGGAGAATT

### 2.8 Real‐time PCR

Total RNA from cultured chondrocytes was extracted and then reverse‐transcribed into cDNA. The expression levels of different genes were determined by real‐time PCR analysis using the FS Universal SYBR Green Real Master (Roche) as previously described.^20^ The results were analysed using LightCycler 96 Software. After analysis using the 2^−ΔΔCt ^method, data were normalized to GAPDH expression. Primers were designed according to the conserved regions of white‐tailed deer, human, cattle and sheep mRNA sequences and listed in Table 2.

**Table 2:** Primers used in this study

Gene	Forward primer	Reverse primer	Size (bp)
Ccnd1	GCGCAGACCTTCGTTGCCCT	GCCGTTGGCGCTTCCCAGAT	123
Ccnd2	AACACCGATGTGGATTGCC	GGAGAGAGCGGATTGGACG	211
Ccnd3	ATTGGGAGGTGCTGGTCTTG	TGTGGCAATCATGGATGGGG	200
Ccne1	ACTTCTGTACCCACACGCTG	TTGCTCGCATTTTAGGCTGC	194
Cdk2	GCTCACTGGCATTCCTCTTC	ACCCATCTGCGTTGATAAGC	134
Cdk4	AGTGACCCTGGTGTTTGAGC	GCAGTTGGCATGAAGGAAAT	142
Cdk6	TCGTGGAAGTTCAGATGTCG	TTGGTTGAGGGGATTTTGAG	128
Col X	ATCCCCGGCCCAGCTGGAAT	GGGAGGCCCCTCTCACCTGG	179
Runx2	TCAGAACCCACGGCCCTCCC	GACAGCGGCGTGGTGGAGTG	177
Alpl	GGAAGGGGGCAGGATTGAC	GGTGTACCCGCCAAAGGTAA	175
Notch1	AACCGTAGCTCCTGAGAGCA	AGAGTCTGATCGTGCCCACT	116
Notch2	TCGCTTCCAGTGTCTGTGTC	ACACTTTGCCCCATTCAGAC	100
Shh	GTGATCCTTGCTTCCTCGCT	TGTCGGGGTTGTAATTGGGG	223
Smo	GTTCGGACAGACAACCCCAA	GATTCGAGTTCCGCCAGTCA	190
Gli1	CTGAGCCTTATGGAGCTAGA	AATGTTCAAGACGAGGACAC	207
Gli2	GCACCACCCCCTCAGACTAT	AGAGTGGGGAGATGGACAGC	207
Gli3	ACCATACGTCTGTGAGCACG	ATGTTTCCGGAGGGAGCTTG	160
Foxa1	CTTTCAAGCGCAGCTATCCT	TCGCTCAGTGTGAGCATCTT	103
Foxa2	TCATGTCGTCAGAGCAGCAG	CCCCTGGTAGTAGGAGGTGT	200
Foxa3	GGGCTCGGTGAAGATGGAG	GTCATGTAGGAGTTGAGGGGG	120
GAPDH	GAAGGGTGGCGCCAAGAGGG	GGGGGCCAAGCAGTTGGTGG	142

The article "Function and regulation of transforming growth factor β1 signalling in antler chondrocyte proliferation and differentiation" was published in 2019. Journal: Cell Prolif.

### 2.9 Statistical analysis

All the experiments were independently repeated at least three times. The significance of difference was analysed by one‐way ANOVA or independent samples *t* test using the SPSS software program (SPSS Inc). The differences were considered significant at *P* < 0.05.

## 3 RESULTS

### 3.1 TGFβ1, TGFBR1 and TGFBR2 expression in antler cartilage

To examine the expression of TGFβ1, TGFBR1 and TGFBR2 in antler cartilage, immunofluorescence was performed. The results showed that TGFβ1, TGFBR1 and TGFBR2 were highly expressed in antler chondrocytes (Figure 1A).

**Figure 1:** Immunofluorescence analysis of TGFβ1, TGFBR1 and TGFBR2 expression in antler cartilage. Bar = 60 μm

### 3.2 Effects of TGFβ1 signalling on the proliferation and cell cycle of antler chondrocytes

MTS results showed that rTGFβ1 significantly enhanced the proliferative activity of antler chondrocytes, whereas addition of TGFβ1 receptor inhibitor SB431542 impeded this enhancement (Figure 2A). Similarly, flow cytometry analysis revealed that rTGFβ1 accelerated the progression of cell cycle from G1 to S phase, whereas SB431542 significantly slowed this progression (Figure 2B‐C). To further elucidate the molecular basis for the proliferative role of TGFβ1, we examined its regulation on the expression of cyclin D1 (Ccnd1), Ccnd2, Ccnd3, Ccne1, cyclin‐dependent kinase 2 (Cdk2), Cdk4 and Cdk6. The results showed that rTGFβ1 increased the expression of Ccnd1, Ccnd2, Ccnd3, Ccne1, Cdk2, Cdk4 and Cdk6 in antler chondrocytes, while SB431542 abolished the rTGFβ1‐induced stimulation of these genes (Figure 2D,E).

**Figure 2:** Effects of TGFβ1 signalling on the proliferation and cell cycle of antler chondrocytes. A, Effects of TGFβ1 signalling on antler chondrocyte proliferation. After treatment with rTGFβ1 in the absence or presence of receptor inhibitor SB431542 and Smad3 inhibitor SIS3, MTS assay was performed. Data are shown mean ± SEM. Asterisks denote significance (*P* < 0.05). B and C, Effects of TGFβ1 signalling on cell cycle of antler chondrocytes. D and E, Effects of TGFβ1 signalling on the expression of Ccnd1, Ccnd2, Ccnd3, Ccne1, Cdk2, Cdk4 and Cdk6

Western blot analysis showed that exogenous rTGFβ1 enhanced the expression of Smad3 and p‐Smad3, but this enhancement was reversed by SB431542 (Figure 3A,B). Administration of Smad3 inhibitor SIS3 weakened the induction of rTGFβ1 on chondrocyte proliferation and expression of Ccnd1, Ccnd2, Ccnd3, Ccne1, Cdk2, Cdk4 and Cdk6, and delayed G1/S phase transition elicited by rTGFβ1 (Figure 2A‐E).

The article "Function and regulation of transforming growth factor β1 signalling in antler chondrocyte proliferation and differentiation" was published in 2019. Journal: Cell Prolif.

**Figure 3:** TGFβ1 signalling regulates antler chondrocyte differentiation. A and B, Western blot analysis of Smad3 and p‐Smad3 protein expression after treatment with rTGFβ1 in the absence or presence of SB431542. C‐E, Col X, Runx2 and Alpl expression after treatment with rTGFβ1 for 3, 6, 12 and 24 h. F, SB431542 or SIS3 abrogated the effects of rTGFβ1 on the expression of Col X, Runx2 and Alpl

### 3.3 Effects of TGFβ1 signalling on antler chondrocyte differentiation

To determine the role of TGFβ1 signalling in antler chondrocyte differentiation, we investigated its influence on the expression of type X collagen (Col X), runt‐related transcription factor 2 (Runx2) and alkaline phosphatase (Alpl), the well‐known markers for hypertrophic chondrocytes.^22^, ^23^ The results indicated that Col X, Runx2 and Alpl mRNA levels were increased in a time‐dependent manner after rTGFβ1 treatment, but this increase was abrogated by SB431542 and SIS3 (Figure 3C‐F).

### 3.4 Notch signalling mediates the effects of TGFβ1 on antler chondrocyte proliferation and differentiation

Notch signalling is important for chondrocyte proliferation and differentiation.^14^, ^15^, ^16^ Our previous studies demonstrated that Notch1 and Notch2 mRNA levels were abundant in antler chondrocytes.^17^ Exposure to rTGFβ1 caused an increase for Notch1 and Notch2 mRNA, whereas SB431542 and SIS3 blocked this increase (Figure 4A), implying that Notch pathway may be downstream of TGFβ1 signalling. Indeed, inhibition of Notch signalling by DAPT hindered the stimulation of rTGFβ1 on antler chondrocyte proliferation and expression of Ccnd1, Ccnd2, Ccnd3, Ccne1, Cdk2, Cdk4 and Cdk6, and deferred the transition of cell cycle from G1 into S phase caused by rTGFβ1 (Figure 4B‐F). Subsequently, we examined the role of Notch signalling in TGFβ1‐mediated chondrocyte differentiation. The results showed that DAPT effectively decreased the promotion of Col X, Runx2 and Alpl by rTGFβ1 (Figure 4G).

**Figure 4:** Notch signalling mediates the effects of TGFβ1 on antler chondrocyte proliferation and differentiation. A, Effects of TGFβ1 signalling on Notch1 and Notch2 expression. B, Notch signalling mediated the effects of TGFβ1 on antler chondrocyte proliferation. After treatment with Notch signalling inhibitor DAPT and addition of rTGFβ1, MTS assay was performed. C and D, Notch signalling mediated the effects of TGFβ1 on cell cycle of antler chondrocytes. E and F, Notch signalling mediated the effects of rTGFβ1 on the expression of Ccnd1, Ccnd2, Ccnd3, Ccne1, Cdk2, Cdk4 and Cdk6. G, Notch signalling mediated the effects of TGFβ1 on the expression of Col X, Runx2 and Alpl

The article "Function and regulation of transforming growth factor β1 signalling in antler chondrocyte proliferation and differentiation" was published in 2019. Journal: Cell Prolif.

### 3.5 Shh signalling mediates the effects of TGFβ1 on antler chondrocyte proliferation and differentiation

In antler chondrocytes, rTGFβ1 raised the expression of Shh, Smo, Gli1, Gli2 and Gli3, while SB431542 and SIS3 attenuated the effects of rTGFβ1 on these genes (Figure 5A,B). Supplementation with Smo antagonist cyclopamine, which also blocked hedgehog signalling, ablated the regulation of rTGFβ1 on chondrocyte proliferation and the expression of Ccnd1, Ccnd2, Ccnd3, Ccne1, Cdk2, Cdk4 and Cdk6, and weakened G1/S phase transition induced by rTGFβ1 (Figure 5C‐G). Moreover, addition of rShh effectively ameliorated the impairment of SB431542 and SIS3 on antler chondrocyte proliferation, rescued cell cycle progression with an increased accumulation of cells in S phase and abolished the inhibition of SB431542 or SIS3 on the expression of Ccnd1, Ccnd2, Ccnd3, Ccne1, Cdk2, Cdk4 and Cdk6 (Figure 6A‐J).

**Figure 5:** Shh signalling mediates the effects of TGFβ1 on antler chondrocyte proliferation. A and B, Effects of TGFβ1 signalling on the expression of Shh, Smo, Gli1, Gli2 and Gli3. C, Shh signalling mediated the effects of TGFβ1 on antler chondrocyte proliferation. After treatment with Smo antagonist cyclopamine, which could also blocked hedgehog signalling, and addition of rTGFβ1, MTS assay was performed. Cyc, cyclopamine. D and E, Shh signalling mediated the effects of TGFβ1 on cell cycle of antler chondrocytes. F and G, Shh signalling mediated the effects of TGFβ1 on the expression of Ccnd1, Ccnd2, Ccnd3, Ccne1, Cdk2, Cdk4 and Cdk6

**Figure 6:** Shh rescues the effects of SB431542 and SIS3 on antler chondrocyte proliferation. A, Exogenous rShh restored the effects of SB431542 on antler chondrocyte proliferation. After treatment with SB431542 and addition of rShh, MTS assay was performed. B and C, Exogenous rShh rescued the effects of SB431542 on cell cycle of antler chondrocytes. D and E, Exogenous rShh reversed the repression of SB431542 on the expression of Ccnd1, Ccnd2, Ccnd3, Ccne1, Cdk2, Cdk4 and Cdk6. F, Exogenous rShh rescued the effects of SIS3 on antler chondrocyte proliferation. G and H, Exogenous rShh restored the effects of SIS3 on cell cycle of antler chondrocytes. I and J, Exogenous rShh improved the regulation of SIS3 on the expression of Ccnd1, Ccnd2, Ccnd3, Ccne1, Cdk2, Cdk4 and Cdk6

In addition, we examined the role of Notch signalling in TGFβ1‐mediated chondrocyte differentiation. After treatment with Shh siRNA or Smo antagonist cyclopamine and addition of rTGFβ1, the expression levels of Col X, Runx2 and Alpl were obviously lessened compared with rTGFβ1 treatment alone followed by the down‐regulation of Gli1, Gli2 and Gli3 (Figure 7A‐D). Inhibition of Gli transcription factors by Gli1 antagonist GANT58 or corresponding siRNA decreased the induction of Col X, Runx2 and Alpl by rTGFβ1 (Figure 7E‐H). Further analysis showed that rShh improved the suppressive effects of SB431542 or SIS3 on Smo, Gli1, Gli2 and Gli3, and recovered antler chondrocyte differentiation as indicated by the elevated mRNA levels for Col X, Runx2 and Alpl (Figure 7I‐L).

The article "Function and regulation of transforming growth factor β1 signalling in antler chondrocyte proliferation and differentiation" was published in 2019. Journal: Cell Prolif.

**Figure 7:** Shh signalling mediates the effects of TGFβ1 on antler chondrocyte differentiation. A, Shh siRNA impeded the effects of TGFβ1 on the expression of Col X, Runx2 and Alpl. NC, negative control; siShh, Shh siRNA. B, Smo mediated the effects of TGFβ1 on the expression of Col X, Runx2 and Alpl. C, Shh siRNA impeded the effects of TGFβ1 on the expression of Gli1, Gli2 and Gli3. D, Smo mediated the effects of TGFβ1 on the expression of Gli1, Gli2 and Gli3. E, Gli antagonist GANT58 blocked the effects of TGFβ1 on the expression of Col X, Runx2 and Alpl. F‐H, Gli1, Gli2 and Gli3 siRNA impeded the effects of TGFβ1 on the expression of Col X, Runx2 and Alpl. siGli1, Gli1 siRNA; siGli2, Gli2 siRNA; siGli3, Gli3 siRNA. I and J, Exogenous rShh reversed the effects of SB431542 and SIS3 on the expression of Smo, Gli1, Gli2 and Gli3. K and L, Exogenous rShh ameliorated the regulation of SB431542 and SIS3 on the expression of Col X, Runx2 and Alpl

### 3.6 Notch pathway mediates TGFβ1‐induced activation of Shh signalling in antler chondrocytes

As stated above, TGFβ1 activated Notch and Shh signalling. In antler chondrocytes, Notch signalling was upstream of Shh pathway.^17^ Based on these observations, we hypothesized that TGFβ1 modulated Shh signalling via Notch pathway. To test this hypothesis, we treated antler chondrocytes with Notch signalling inhibitor DAPT, supplemented exogenous rTGFβ1 and then analysed the expression of Shh, Smo, Gli1, Gli2 and Gli3. The results revealed that DAPT might counteract the induction of rTGFβ1 on Shh, Smo, Gli1, Gli2 and Gli3 (Figure 8A,B).

**Figure 8:** TGFβ1 activates Shh signalling through Notch pathway and regulates antler chondrocyte differentiation via Foxa. A and B, DAPT attenuated the effects of TGFβ1 on the expression of Shh, Smo, Gli1, Gli2 and Gli3. C, Effects of TGFβ1 signalling on the expression of Foxa1, Foxa2 and Foxa3. D‐F, Foxa1, Foxa2 and Foxa3 siRNA impeded the effects of TGFβ1 on the expression of Col X, Runx2 and Alpl. siFoxa1, Foxa1 siRNA; siFoxa2, Foxa2 siRNA; siFoxa3, Foxa3 siRNA

### 3.7 TGFβ1 signalling regulates antler chondrocyte differentiation through Foxa

It is well known that Foxa transcription factors are critical for chondrocyte differentiation.^19^ In antler chondrocytes, rTGFβ1 enhanced the expression of Foxa1, Foxa2 and Foxa3, but these effects were attenuated by SB431542 and SIS3 (Figure 8C). Furthermore, silencing of Foxa1, Foxa2 or Foxa3 via their corresponding siRNA failed to induce the expression of Col X, Runx2 and Alpl (Figure 8D‐F).

The article "Function and regulation of transforming growth factor β1 signalling in antler chondrocyte proliferation and differentiation" was published in 2019. Journal: Cell Prolif.

### 3.8 Notch and Shh signalling mediate the regulation of Foxa by TGFβ1 in antler chondrocytes

As described above, TGFβ1 was upstream of Notch and Shh signalling which controlled the expression of Foxa transcription factors. Therefore, we analysed whether Notch and Shh signalling might mediate the regulation of Foxa by TGFβ1. Blockage of Notch signalling by DAPT alleviated the up‐regulation of Foxa1, Foxa2 and Foxa3 induced by rTGFβ1 (Figure 9A). Consistently, after treatment with Shh siRNA or Smo antagonist cyclopamine, rTGFβ1 failed to augment the expression of Foxa1, Foxa2 and Foxa3 (Figure 9B,C). Meanwhile, suppression of Gli transcription factors by GANT58 or corresponding siRNA weakened the rTGFβ1‐mediated induction of Foxa1, Foxa2 and Foxa3 (Figure 9D‐G). Moreover, rShh reversed the regulation of SB431542 or SIS3 on the expression of Foxa1, Foxa2 and Foxa3 (Figure 9H,I).

**Figure 9:** Notch and Shh signalling mediate the regulation of TGFβ1 on Foxa in antler chondrocytes. A, Notch signalling mediated the effects of TGFβ1 on the expression of Foxa1, Foxa2 and Foxa3. B, Shh siRNA prevented the effects of TGFβ1 on the expression of Foxa1, Foxa2 and Foxa3. C, Smo mediated the effects of TGFβ1 on the expression of Foxa1, Foxa2 and Foxa3. D, GANT58 blocked the regulation of TGFβ1 on the expression of Foxa1, Foxa2 and Foxa3. E‐G, Gli1, Gli2 and Gli3 siRNA impeded the effects of TGFβ1 on the expression of Foxa1, Foxa2 and Foxa3. H and I, Exogenous rShh ameliorated the regulation of SB431542 and SIS3 on the expression of Foxa1, Foxa2 and Foxa3

## 4 DISCUSSION

The diagnosis and treatment of bone disease are difficult and have become hot topics in medical research. Chondrocytes are produced by mesenchymal stem cells, which undergo proliferation followed by differentiation, and eventually develop into bone during skeletogenesis.^24^, ^25^ As a unique bony organ, antler re‐growth is characterized by the non‐cancerous rapid proliferation and differentiation of chondrocytes, which are crucial for fracture healing, osteoarthritis and skeletal dysplasia; thus, this is a good model for studying cartilage development and bone diseases.^2^, ^17^ To date, the molecular mechanisms controlling the proliferation and differentiation of antler chondrocytes are not well understood. Here, we provide evidence of the role of TGFβ1 signalling in antler chondrocyte proliferation and differentiation, and explore its interaction with Notch, Shh signalling and Foxa.

The article "Function and regulation of transforming growth factor β1 signalling in antler chondrocyte proliferation and differentiation" was published in 2019. Journal: Cell Prolif.

It has previously been shown that TGFβ1 plays a role in inducing chondrocyte proliferation and maintaining phenotypic stability.^5^, ^26^ Cell proliferation is dependent on four distinct phases of the cell cycle (G0/G1, S, G2 and M), which are regulated by a complex interplay of cyclins and Cdks.^27^, ^28^ Our study demonstrated that rTGFβ1 promoted cell proliferation, accelerated cell cycle transition from G1 to S phase and increased the expression of Ccnd1, Ccnd2, Ccnd3, Ccne1, Cdk2, Cdk4 and Cdk6. Similarly, mice lacking Ccnd1 showed dwarfism along with the reduced chondrocyte proliferation.^29^ In addition, chondrocyte differentiation was associated with gradual increase of hypertrophic chondrocyte markers.^30^ The current evidence indicated that TGFβ1 could stimulate the expression of Col X, Runx2 and Alpl, well‐known markers for hypertrophic chondrocytes. Similar stimulation of chondrocyte differentiation was observed when TGFβ1 was injected into the knee joints of mice or rabbits.^31^, ^32^ Thus, the above results led us to further investigate the mechanism of TGFβ1 in stimulating chondrocyte proliferation and differentiation. TGFβ1 acts through its receptor TGFBR1, which binds to TGFBR2, and subsequently recruits other signalling molecules including receptor‐associated Smad3.^33^ In antler chondrocytes, TGFβ1 could activate the expression of Smad3, while receptor inhibitor SB431542 impeded this activation. As shown in Meckel's cartilage of TGFBR2^fl/fl^, cell proliferation activity was significantly reduced.^34^ Moreover, addition of Smad3 inhibitor SIS3 slowed the proliferation and differentiation of antler chondrocytes induced by rTGFβ1. Targeted disruption of Smad3 exon 8 or deficiency of Smad2/3 led to skeletal abnormalities along with the aberrant chondrocyte proliferation and differentiation.^11^, ^35^ Collectively, TGFβ1 signalling plays an important role in promoting the proliferation and differentiation of antler chondrocytes.

It is well known that after binding to TGFBR1/2, TGFβ1 induces Smad3 phosphorylation and further activates related downstream genes.^26^ Notch and TGFβ1 signalling are important for controlling cell differentiation during cartilage formation, for example, TGFβ1 signalling regulates mouse hepatic stellate cell differentiation via Notch pathway.^36^ Moreover, Notch and TGFβ signalling are known to converge in the regulation of several other differentiation events, such as endothelial, pancreas and neural development.^37^ These findings prompted us to investigate the relationship between TGFβ1 and Notch signalling in chondrocyte proliferation and differentiation. In antler chondrocytes, DAPT effectively attenuated the regulation of TGFβ1 on chondrocyte proliferation and differentiation, indicating that TGFβ1 was upstream of Notch signalling.

The article "Function and regulation of transforming growth factor β1 signalling in antler chondrocyte proliferation and differentiation" was published in 2019. Journal: Cell Prolif.

Shh is known to play a critical role in normal chondrocyte proliferation and differentiation.^38^ Loss of Shh led to developmental defects in Meckel's cartilage and mandibular hypoplasia.^39^ It is generally accepted that Shh activates Smo, which promotes Gli protein transport into the nucleus to facilitate the transcription of target gene.^40^ Further studies demonstrated that Notch pathway was upstream of Shh signalling, and addition of exogenous rShh rescued the delayed onset of DAPT on chondrocyte proliferation and differentiation.^17^ Similar results were obtained in neuroepithelial cells, where activation of Notch enhanced the activity of Shh, which increased Smo accumulation and induced the elevation of Gli3 levels.^41^ Furthermore, TGFβ1 may affect the expression of Shh and Gli1 during chondrogenic differentiation of MSCs.^18^ More importantly, the present study provided insights into the relationship between TGFβ1 and Shh signalling in antler chondrocytes. Knockout of Shh or addition of Smo antagonist cyclopamine attenuated the induction of TGFβ1 on chondrocyte proliferation and differentiation, whereas exogenous rShh rescued the delayed onset of chondrocyte proliferation and differentiation elicited by SB431542 and SIS3, indicating that TGFβ1 pathway was upstream of Shh signalling. In addition, high concentrations of Shh induced the expression of Foxa2.^42^ Previous research has shown that Foxa transcription factors act as downstream targets of Shh signalling to regulate antler chondrocyte proliferation and differentiation.^17^ Moreover, transfection with siRNA targeting Foxa reduced the induction of rTGFβ1 on Col X, Runx2 and Alpl, confirming that TGFβ1 signalling regulated antler chondrocyte differentiation via Foxa transcription factors. Further analysis evidences that Shh signalling plays an important role in the crosstalk between TGFβ1 and Foxa transcription factors.

In summary, this study reveals that TGFβ1 signalling may induce the proliferation and differentiation of antler chondrocytes through Notch‐Shh‐Foxa pathway (Figure 10).

**Figure 10:** Schematic diagram shows the interplay of TGFβ1, Notch, Shh signalling and Foxa in antler chondrocyte proliferation and differentiation. TGFβ1 signalling could induce the proliferation and differentiation of antler chondrocytes through Notch‐Shh‐Foxa pathway

## CONFLICT OF INTEREST

The authors declare that there is no conflict of interest.
